The article "Fenretinide Corrects the Imbalance between Omega-6 to Omega-3 Polyunsaturated Fatty Acids and Inhibits Macrophage Inflammatory Mediators via the ERK Pathway" was published in 2013. Journal: PLoS One.

# Fenretinide Corrects the Imbalance between Omega-6 to Omega-3 Polyunsaturated Fatty Acids and Inhibits Macrophage Inflammatory Mediators via the ERK Pathway

**DOI:** 10.1371/journal.pone.0074875

**Published:** 2013-09-12

**Authors:** Claude Lachance, Gabriella Wojewodka, Tom A. A. Skinner, Claudine Guilbault, Juan B. De Sanctis, Danuta Radzioch

**Affiliations:** 1 McGill University, Department of Medicine and Department of Human Genetics, McGill University Health Center Research Institute, Montreal, Quebec, Canada; 2 Central University of Venezuela, Institute of Immunology, Caracas, Venezuela; The Ohio State University, United States of America

## Abstract

We previously identified Fragile X-related protein 1 (FXR1) as an RNA-binding protein involved in the post-transcriptional control of TNF and other cytokines in macrophages. Macrophages derived from FXR1-KO mice overexpress several inflammatory cytokines including TNF. Recently, we showed that fenretinide (4HPR) is able to inhibit several inflammatory cytokines in the lungs of cystic fibrosis mice, which also have abnormal immune responses. Therefore, we hypothesized that 4HPR might also be able to downregulate excessive inflammation even in macrophages with ablated FXR1. Indeed, our results demonstrate that 4HPR inhibited the excessive production of inflammatory mediators, including TNF, IL-6, CCL2 and CCL-5 in LPS-stimulated FXR1-KO macrophages, by selectively inhibiting phosphorylation of ERK1/2, which is naturally more phosphorylated in FXR1-KO cells. We also found that LPS stimulation of FXR1-KO macrophages led to significantly higher ratio of arachidonic acid/docosahexaenoic acid than observed in FXR1-WT macrophages. Interestingly, treatment with 4HPR was associated with the normalization of arachidonic acid/docosahexaenoic acid ratio in macrophages, which we found to impact phosphorylation of ERK1/2. Overall, this study shows for the first time that 4HPR modulates inflammatory cytokine expression in macrophages by correcting a phospholipid-bound fatty acid imbalance that impacts the phosphorylation of ERK1/2.

## Introduction

Activated macrophages play important roles in the regulation of inflammatory responses by releasing inflammatory cytokines and chemokines, which in turn stimulate and attract other cells of the immune system [1]. The release of inflammatory cytokines and chemokines is tightly controlled both spatially and temporally. Post-transcriptional regulation of cytokines and chemokines represents an important mechanism to effectively and rapidly regulate gene expression and hence immune responses [2]. Structures such as the AU-rich elements (AREs), which are present in the 3′-untranslated region of many mRNAs, enable the regulation of mRNA turnover and translation rate through their interactions with ARE-RNA binding proteins (RBPs). ARE-RBPs such as tristetraprolin (TTP) [3] and ARE/poly-(U)-binding/degradation factor 1 (AUF1) [4] have been found to destabilize mRNAs such as tumor necrosis factor (TNF) mRNA. Conversely, HuR is an ARE-RBP that has been described as a positive regulator of mRNA stability [5], [6]. The T-cell internal antigen-1 (TIA-1) and TIA-1-related protein (TIAR) are closely related proteins that have been found to inhibit the translation of TNF mRNA in macrophages [7]. We previously showed that Fragile X-related protein 1 (FXR1) is also capable of binding to the AREs of TNF mRNA, downregulating its expression at the post-transcriptional level [8].

The article "Fenretinide Corrects the Imbalance between Omega-6 to Omega-3 Polyunsaturated Fatty Acids and Inhibits Macrophage Inflammatory Mediators via the ERK Pathway" was published in 2013. Journal: PLoS One.

AREs and RBPs regulate mRNA stability and/or translational processing in response to stress stimuli such as lipopolysaccharide (LPS). The mechanisms involved in this regulation are dependent on mitogen-activated protein kinases (MAPKs). For instance, it is well established that the p38 MAPK pathway is involved in the regulation of cyclooxygenase-2 (Cox-2) mRNA stability [9], [10]. MAPKs are well-conserved, signaling proteins which are activated in response to stress and stimulation with various bacterial products [11]. Two members of the MAPK family, p38 MAPK and extracellular signal-regulated kinase (ERK), are particularly important in the regulation of cytokine gene expression in macrophages [12], [13]. Interactions between ERK1/2, p38 MAPK and ARE-RBPs have been documented but are not fully understood. For example, the p38 signal transduction pathway can control the expression and post-translational modification of TTP, which is implicated in destabilizing TNF mRNA [14]. Subsequently, it was demonstrated that the activities of both ERK and p38 MAPK are required for inhibition of TTP function and stabilization of TNF mRNA [15].

Interestingly, Lo and colleagues reported that LPS-stimulated macrophages grown in the presence of eicosapentaenoic acid had reduced ERK1/2 phosphorylation [16]. It was also shown that production of TNF by macrophages can be modified by oxidized 1-palmitoyl-2-arachidonoyl-*sn*-glycero-3-phosphorylcholine (PAPC) and that oxidized PAPC alters the p38 MAPK phosphorylation pathway [17]. Thus, fatty acids can exert a certain level of control on gene expression via MAPK pathways. Recently, our studies showed that treatment with fenretinide (*N*-(4-hydroxyphenyl) retinamide (4HPR)), a vitamin A derivative, is able to both downregulate the production of arachidonic acid (AA), a pro-inflammatory omega-6 polyunsaturated fatty acid, and to increase levels of omega-3 polyunsaturated docosahexaenoic acid (DHA), which has an anti-inflammatory effect [18], [19]. We also showed that treatment with 4HPR is able to inhibit certain inflammatory cytokines in the lungs of cystic fibrosis transmembrane conductance regulator (*Cftr*)-knockout mice with chronic inflammatory lung disease [20]. Therefore, we postulated that 4HPR might also be able to normalize the excessive production of inflammatory cytokines caused by the deletion of the *Fxr1* gene. In this study, we assessed the effect of 4HPR treatment on gene expression, regulation of signaling molecule activation, and phospholipid-bound fatty acid composition in macrophages. Our findings shed new light on the possible molecular mechanism responsible for the excessive production of inflammatory cytokines by *Fxr1*-knockout (FXR1-KO) macrophages and identify pharmacological targets for the selective inhibition of several AU-rich genes regulated post-transcriptionally by FXR1.

The article "Fenretinide Corrects the Imbalance between Omega-6 to Omega-3 Polyunsaturated Fatty Acids and Inhibits Macrophage Inflammatory Mediators via the ERK Pathway" was published in 2013. Journal: PLoS One.

## Materials and Methods

### Reagents

Ultra-pure LPS from *Escherichia coli* 0111:B4 was obtained from Invivogen (San Diego, CA). The ERK1/2 inhibitors UO126 and PD98059 were purchased from Calbiochem (Gibbstown, NJ). Phospho-p44/p42 MAP Kinase (Thr202/Tyr204), p44/p42 MAP Kinase, phospho-p38 MAP Kinase (Thr180/Tyr182), and p38 MAP Kinase antibodies were purchased from Cell Signaling (Danvers, MA). Monoclonal anti-mouse TNF antibody and recombinant murine TNF were obtained from R&D (Minneapolis, MN). Arachidonic acid (AA), docosahexaenoic acid (DHA), and butylated hydroxyanisole (BHA) were purchased from Sigma-Aldrich (St-Louis, MO). The synthetic retinoid, 4HPR powder [*N*-(4-hydroxyphenyl) retinamide] was generously provided by Dr. R. Smith (NIH) and resuspended in 95% ethanol at an initial concentration of 2 mg/ml. Following reconstitution, it was protected from light and kept at −20°C before its addition to cell culture medium.

### Cell Culture

FXR1-KO and FXR1-wildtype (FXR1-WT) macrophage cell lines were derived from the bone marrow of caesarean section-delivered *Fxr1^−/−^* and *Fxr1* ^+/+^ mice, as previously described [8]. Cells were grown in Dulbecco's modified Eagle's medium (Invitrogen, Burlington, Ontario, Canada) supplemented with 6% heat-inactivated fetal bovine serum (Wisent, Saint-Bruno, Québec, Canada), 100 U/ml penicillin (Invitrogen), and 100 µg/ml streptomycin (Invitrogen) and incubated at 37°C and 5% CO_2_.

Cells were plated in 6-well or 24-well plates at a concentration of 2.5×10^5^ cells/ml for 2 h, and thereafter medium was removed and replaced with fresh medium containing either 0.625 µM of 4HPR, 100 nM of AA, or 100 nM of DHA. Cells were allowed to grow for 21 h and then medium was replaced with fresh medium containing the same initial concentration of previously added 4HPR, AA, or DHA, and 5 µM of ERK1/2 inhibitors were added for 1 h where appropriate. Cells were then stimulated with 50 ng/ml of LPS for 3 h in all experiments, except in assays evaluating the activation of MAPK signaling pathways where the stimulation time was 30 min. All experiments included untreated and/or unstimulated negative control wells.

The article "Fenretinide Corrects the Imbalance between Omega-6 to Omega-3 Polyunsaturated Fatty Acids and Inhibits Macrophage Inflammatory Mediators via the ERK Pathway" was published in 2013. Journal: PLoS One.

### Cell Treatment with Fatty Acids

The 100 mM stock solutions of AA or DHA solutions were prepared in ethanol. The stock solutions of AA or DHA were then complexed with BSA at a molar ratio of 2.5∶1. The AA- and DHA-BSA mixtures were then diluted in media (1000 times) to a final concentration of 100 nM of the fatty acids and added to a cell suspension in 24-well Costar plates. Control cells were incubated with the same amount of vehicle and the same about of BSA as the treated cells. Neither DHA-BSA, AA-BSA nor vehicle control containing equivalent amounts of BSA had any effect on cell viability.

### Analysis of Phospholipid-Esterified Fatty Acids from FXR1-WT and KO Macrophage Cell Lines

A total of 5×10^7^ FXR1-WT or KO cells were seeded in two 175 cm^2^ flasks (Sarstedt, Montreal, Qc, Canada) and were treated as indicated in the previous section. Macrophages were stimulated with 50 ng/ml of LPS for 3 h or left unstimulated. Cells were subsequently harvested and centrifuged at 300×*g* for 5 min. The cell pellet was washed once with phosphate buffered saline (PBS) (Invitrogen) and then resuspended immediately with 1 ml of BHA solution (1 mM BHA: 2 vol. chloroform: 1 vol. methanol) to extract lipids from the macrophages and to prevent lipid oxidation. Samples were stored at −80°C until analysis.

Lipids were extracted according to the Folch method [21]. Briefly, one volume of cold water is added to the mixture and samples are mixed for 90 min at 4°C. The organic phase is collected to which diethyl ether is added to remove any leftover protein contamination. The fraction is dried and resuspended in 100 µl of chloroform. Fatty acids were identified by thin layer chromatography extraction performed as described previously [19], [20], [22]. Briefly, diazomethane was used to esterify the released fatty acids [23] and the esters were identified by GC/MS (Hewlett Packard 5880A, WCOT capillary column (Supelco-10, 35 m×0.5 mm, 1 µM thick)) using commercial standards (Sigma-Aldrich). Protein concentrations were assessed using the bicinchoninic acid assay (Pierce Biotechnology, Rockford, IL).

### Lipid Peroxidation Analysis

Lipid peroxidation was measured fluorometrically using 2-thiobarbituric acid-reactive substances (TBARS) as surrogate for malonyldealdehyde, the end product of lipid peroxidation [24], [25]. Briefly, plasma samples were mixed with 8.1% sodium dodecyl sulfate, 20% acetic acid and 0.8% 2-thiobarbituric acid. After vortexing, samples were incubated for 1 h at 95°C after which butanol-pyridine at 15∶1 (v/v) ratio was added. The mixture was shaken for 10 min and then centrifuged. The butanol-pyridine layer was measured fluorometrically at 552 nm after excitation at 515 nm (Shimadzu, Japan). The results are expressed in nmole TBARS/mg of protein which reflects the levels of malonyldealdehyde in the samples as well as any other thiobarbituric acid reactive substances, if any should have arisen during the assay [26].

The article "Fenretinide Corrects the Imbalance between Omega-6 to Omega-3 Polyunsaturated Fatty Acids and Inhibits Macrophage Inflammatory Mediators via the ERK Pathway" was published in 2013. Journal: PLoS One.

### Nitrotyrosine Analysis

The total amount of 3-nitrotyrosine was determined by ELISA as previously described by Montes de Oca *et al* [27] using previously characterized antibodies [28]. Antibodies (mouse IgG monoclonal, polyclonal against nitrotyrosine and polyclonal goat anti-rabbit IgG-peroxidase) were from Upstate Biotechnology (Lake Placid, NY). The quantification of nitrotyrosine was performed using a standard curve with known concentrations of nitrotyrosine from chemically modified bovine serum albumin. The sensitivity of the assay was 50 pg/ml.

### TNF ELISA

The amount of secreted TNF in supernatants of stimulated macrophages was determined using a sandwich TNF ELISA assay. Following treatment, cell culture supernatants were harvested and centrifuged at 100×*g* to remove floating cells and debris. Plates (96-well, Nalge Nunc, Rochester, NY) were coated overnight at 4°C with a hamster anti-TNF monoclonal antibody, blocked for 1 h at room temp with 1% bovine serum albumin fraction V (Sigma-Aldrich) in PBS and 0.1% Tween 20 (Fisher, Ottawa, Ontario, Canada), followed by 1 h incubation with the cell culture supernatants or the recombinant murine TNF as the standard. Plates were then incubated for 1 h with a polyclonal rabbit anti-murine TNF antibody followed by 1 h incubation with a horseradish peroxidase-conjugated antibody against rabbit IgG (Bio-Rad, Mississauga, Ontario, Canada). After addition of ABTS reagent mixture (Roche, Laval, Qc, Canada), plates were read at 405 nm. TNF concentrations were calculated based on the standard curve and dilution factor.

### Analysis of Cytokine Protein Expression Using the Luminex 100 LS Platform Assay

The levels of cytokines and chemokines were measured in the supernatants collected from FXR1-KO and FXR1-WT macrophage cell lines stimulated with either 4HPR, AA, DHA, and/or MAPK inhibitors followed by 3 h stimulation with 50 ng/ml of LPS or medium using the Luminex 100 LS platform assay. A multiple cytokine analysis kit (Millipore, Billerica, MA) containing multiplex beads specific for TNF, IL-6, CCL2/MCP-1, and CCL5/RANTES was used. Data were collected using the Luminex-100 LS system with software version 2.3 (Luminex Corporation, Austin, TX) and analyzed using Beadview multiplex data analysis software (Version 1.04; Upstate).

The article "Fenretinide Corrects the Imbalance between Omega-6 to Omega-3 Polyunsaturated Fatty Acids and Inhibits Macrophage Inflammatory Mediators via the ERK Pathway" was published in 2013. Journal: PLoS One.

### Analysis of Gene Expression by Real-Time RT-PCR

Following treatment of FXR1-WT and KO macrophage cell lines, culture medium was removed and cells were washed twice with PBS. Total cellular RNA was extracted using Trizol reagent (Invitrogen) according to manufacturer's instructions. Next, 1 µg of total RNA was reverse-transcribed with QuantiTect reverse transcription kit (Qiagen, Mississauga, Ontario, Canada). The amplification program for the detection of TNF cDNA consisted of an enzyme activation step for 10 min at 95°C, followed by 40 cycles of a denaturing step for 30 s at 95°C, an annealing step for 30 s at 56°C and an extension step for 30 s at 72°C. GAPDH was used as the normalizing gene to compensate for potential differences in the total amount of cDNA. The FXR1-WT unstimulated group was used as reference in steady state level analysis. The primers used for amplification of TNF (forward 5′-AGA CCC TCA CAC TCA GAT CAT CTT C-3′ and reverse 5′-CCT CCA CTT GGT GGT TTG CT-3′) and GAPDH (forward 5′-ATG TGT CCG TCG TGG ATC TGA-3′ and reverse 5′-TTG AAG TCG CAG GAG ACA ACC T-3′) were all tested previously to achieve amplification efficiency between 90 and 100%. The primers sequences were all designed from NCBI GenBank mRNA sequence using the web based software Primerquest from Integrated DNA technologies (http://www.idtdna.com/Scitools/Applications/Primerquest/). The Stratagene MX-4000 sequence detector (Stratagene, La Jolla, CA) was used for amplification of target cDNA of TNF and cDNA of GAPDH for normalization. Quantitation of TNF mRNA expression was calculated using the 2^-ΔΔ*Ct*^ method [29] where ΔΔ*Ct*  =  (*C*_T,Target_ - *C*_T,GADPH_)_sample_ - (*C*_T,Target_ - *C*_T,GADPH_)_calibrator_; the target represents the gene of interest and the calibrator is represented by FXR1-WT untreated (medium) sample.

### Western Blot Analysis

Total cell extracts were prepared from macrophages (1×10^6^ cells) plated in 6-well plates (Corning). After treatments with either 4HPR, AA, DHA, and/or MAPK inhibitors followed by a 30 min stimulation with 50 ng/ml of LPS, medium was removed and cells were washed twice with PBS before lysis with LDS sample buffer (Invitrogen) containing 2.5% 2-mercaptoethanol (Fisher). Next, the samples (10 µg of protein per lane) were separated on NuPAGE 4–12% Bis-Tris gel (Invitrogen). Proteins separated on gels were transferred onto Immobilon-P membranes (Millipore, Mississauga, Ontario, Canada) at 150 mA for 50 min using a semi-dry technique. The membranes were thereafter blocked for 1 h at room temp with a milk solution consisting of 5% PBS/0.1% Tween 20 and stained with a primary antibody overnight at 4°C, followed by an incubation with a secondary horseradish peroxidase-conjugated goat anti-rabbit IgG (Cell Signaling) for 1 h at room temp and Western Lightning™ Chemiluminescence Reagent Plus (Perkin Elmer, Boston, MA) for 1 min. Results were scanned into Photoshop CS2 (Adobe, San Jose, CA) and the intensity of the bands for the corresponding antibodies were analyzed using Imagequant 5.0 (GE healthcare, Piscataway, NJ). The results are expressed as fold induction compared with untreated (medium) FXR1-WT macrophages.

The article "Fenretinide Corrects the Imbalance between Omega-6 to Omega-3 Polyunsaturated Fatty Acids and Inhibits Macrophage Inflammatory Mediators via the ERK Pathway" was published in 2013. Journal: PLoS One.

### Statistical Analysis

All data are expressed as mean ± SEM. Unpaired *t*-test or one way ANOVA followed by a Student-Newman-Keuls secondary analysis were used to compare group mean of normally distributed and equal variance data. If these conditions were not met, a non-parametric ANOVA on ranks statistical test was applied. These statistical tests were performed using Sigmaplot software Version 11 (Systat Software, San Jose, CA). Values of *p*≤0.05 indicate significant differences.

## Results

### Fenretinide Treatment Modulates the Expression of the Inflammatory Cytokine TNF

We previously identified FXR1 as an RNA-binding protein involved in the translational repression of TNF as well as several other cytokines such as IL-1α, IL-1β, IL-6, and GM-CSF expressed by lipopolysaccharide-activated macrophages [8], [30]. We hypothesized that the treatment of macrophages with 4HPR might also be able to diminish excessive production of inflammatory cytokines caused by the ablation of FXR1, an important regulatory RNA-binding protein. To determine whether 4HPR can downregulate LPS-induced TNF secretion by FXR1-KO and FXR1-WT macrophages, cells were pre-treated with 4HPR (0.625 µM) for 21 h and then stimulated with LPS (50 ng/ml) for 3 h. As shown in **Fig. 1**, in response to LPS stimulation, FXR1-KO macrophages secreted more TNF than did FXR1-WT macrophages. Treatment with 4HPR significantly decreased the amount of TNF protein secreted by both FXR1-WT (*p* = 0.005) and FXR1-KO (*p* = 0.004) macrophages compared with the amount of TNF produced by LPS-stimulated macrophages not treated with 4HPR (mock treated).

**Figure 1:** TNF secretion is inhibited by 4HPR in FXR1-WT and KO macrophages following stimulation with the TLR4 ligand LPS. FXR1-WT (▪) and FXR1-KO (□) macrophage cell lines (2.5×10^5^ cells) were untreated or treated with 4HPR (0.625 µM) for 21 h, followed by 3 h stimulation with LPS (50 ng/ml) or Medium alone. Supernatants were harvested and evaluated for TNF protein levels using sandwich ELISA. Results are presented as mean ± SEM of four independent experiments. Differences were analyzed using an unpaired *t*-test and were considered to be significant at *p*≤0.05. * indicates *p*<0.05.

The article "Fenretinide Corrects the Imbalance between Omega-6 to Omega-3 Polyunsaturated Fatty Acids and Inhibits Macrophage Inflammatory Mediators via the ERK Pathway" was published in 2013. Journal: PLoS One.

### Fenretinide Treatment has no Effect on TNF mRNA Steady State Level

To better understand the mechanism(s) by which 4HPR treatment reduced LPS-induced TNF production, we assessed the effect of 4HPR on TNF mRNA steady state level. We found no significant differences in TNF mRNA steady state levels between untreated and 4HPR treated FXR1-WT and KO macrophages, as shown in Table 1A. Although FXR1- KO macrophages showed several-fold higher TNF protein secretion compared with WT cells following 4HPR treatment and LPS stimulation (**Fig. 1**), there were no differences in TNF mRNA steady state levels between FXR1-WT and KO macrophages, as shown in **Table 1B**. These results demonstrate that 4HPR inhibits secretion of TNF protein in macrophages without affecting their TNF mRNA levels, suggesting that 4HPR modulates TNF gene expression in macrophages by another mean.

**Table 1:** TNF mRNA steady state levels in unstimulated or LPS-stimulated FXR1-WT and KO macrophages untreated or treated with 4HPR.

A	Medium	4HPR	*p* values^a^
**FXR1-WT**	1.00±0.35	0.84±0.51	0.999
**FXR1-KO**	2.13±0.34	1.50±0.44	0.976
*p* values^b^	0.159	0.566	

B	LPS	LPS & 4HPR	*p* values^a^
**FXR1-WT**	171.00±37.19	98.98±34.05	0.597
**FXR1-KO**	199.75±72.78	156.00±39.66	0.999
*p* values^b^	1.000	0.819	

Results are expressed as mean ± SEM of TNF mRNA relative expression level using FXR1-WT medium as calibrator. The *p* values were calculated using unpaired *t*-test.

a *p* values refer to Medium versus 4HPR or LPS versus LPS & 4HPR group.

b *p* values refer to FXR1-KO versus FXR1-WT macrophages.

### Excessive Phosphorylation of ERK1/2 in FXR1-KO Macrophages

The involvement of MAP kinases in the regulation of signal transduction pathways leading to the induction of TNF production has been extensively studied [13], [31]–[34]. Previously, we found no significant differences in phospho-p38 MAPK activity between FXR1-WT and FXR1-KO macrophages [8]. In this study, we assessed the phosphorylation of another member of the MAPK family, ERK1/2. As shown in **Fig. 2A**, the level of phospho-ERK1/2 was approximately 4-fold higher in LPS-stimulated FXR1-KO macrophages than in FXR1-WT macrophages (*p* = 0.027). Moreover, basal level of phospho-ERK1/2 was significantly higher in unstimulated FXR1-KO compared with FXR1-WT macrophages (*p* = 0.029). To exclude the possibility that this signaling pathway was activated by macrophage-secreted cytokines, representing a positive feedback loop in culture, macrophages were seeded in 6-well plates and medium was changed every hour for 6 h. Under these conditions, we continued to observe higher phosphorylation of ERK1/2 in non-activated FXR1-KO macrophages than in WT cells (data not shown). This excessive activation of ERK1/2 seems to be selective for this particular MAPK since no significant differences were observed in phospho-p38 kinase regulation between the two macrophage cell lines under unstimulated or LPS-stimulated conditions (*p* = 0.325 and 0.393 respectively) (**Fig. 2B**). These results demonstrate for the first time that the ablation of FXR1 leads to constitutively higher level of phosphorylated ERK1/2, suggesting that this signaling molecule might be directly involved in the FXR1 -dependent regulation of pro-inflammatory gene expression in macrophages.

The article "Fenretinide Corrects the Imbalance between Omega-6 to Omega-3 Polyunsaturated Fatty Acids and Inhibits Macrophage Inflammatory Mediators via the ERK Pathway" was published in 2013. Journal: PLoS One.

**Figure 2:** 4HPR reduces excessive phosphorylation of MAP kinase ERK1/2 in FXR1-KO macrophages. FXR1-WT (▪) and FXR1-KO (□) macrophage cell lines (1×10^6^ cells) were unstimulated (medium) or stimulated for 30 min with LPS (50 ng/ml). Both macrophage cell lines were also treated with 4HPR (0.62 µM) under LPS stimulation conditions. Cells were harvested and kinase phosphorylation levels were analyzed by Western Blot; Total corresponding protein levels (ERK1/2 or p38) were used to normalize differences in loading. (A) Levels of phospho-ERK1/2 and total ERK1/2 MAPK in FXR1-WT and KO cells. (B) Levels of phospho-p38 and total p38 MAPK. Results are presented as mean ± SEM of four independent experiments. Differences were analyzed using an unpaired *t*-test and were considered to be significant at *p*≤0.05. * indicates *p*<0.05.

### Fenretinide Treatment Inhibits Excessive Phosphorylation of ERK1/2 in LPS-Stimulated FXR1-KO Macrophages

Next, we evaluated the effect of 4HPR treatment on the phosphorylation of ERK1/2 in LPS-stimulated macrophages. As shown in **Fig. 2A**, FXR1-WT macrophages treated with 4HPR and then stimulated with LPS for 30 min had significantly less ERK1/2 phosphorylation compared with untreated LPS-stimulated macrophages (*p* = 0.006). Similar results were observed for FXR1-KO macrophages (*p* = 0.015). Interestingly, the treatment of both FXR1-WT and KO macrophages with 4HPR restored ERK1/2 phosphorylation to levels observed in cultured in medium alone (**Fig. 2A**). However, the treatment with 4HPR did not eliminate the initial difference in ERK1/2 phosphorylation observed between the two macrophage types, whether they were stimulated with LPS (*p* = 0.028; **Fig 2A**) or unstimulated (*p* = 0.013; data not shown). Nonetheless, the decrease in ERK1/2 phosphorylation in response to fenretinide treatment was more pronounced in FXR1-KO than WT macrophages (2-fold versus 0.5 fold inhibition respectively).

The article "Fenretinide Corrects the Imbalance between Omega-6 to Omega-3 Polyunsaturated Fatty Acids and Inhibits Macrophage Inflammatory Mediators via the ERK Pathway" was published in 2013. Journal: PLoS One.

We also investigated the effect of 4HPR on p38 phosphorylation (**Fig. 2B**) and we demonstrated that 4HPR did not significantly affect p38 phosphorylation in LPS-stimulated FXR1-WT or KO macrophages (*p* = 0.40 and 0.568 respectively). Taken together, these results indicate that 4HPR mediates inhibition of TNF gene expression via the modulation of the ERK MAPK pathway but not the p38 MAPK pathway.

### Fenretinide Treatment Modulates Expression of Other Inflammatory Proteins in Macrophages

Previously, we showed that FXR1-KO macrophages secreted higher levels of several inflammatory cytokines and chemokines than do FXR1-WT macrophages [30]. Therefore, using the Luminex 100 LS platform assay with cytokine- and chemokine-specific beads, we evaluated the effect of 4HPR on LPS-induced secretion of IL-6, CCL2/MCP-1, and CCL5/Rantes by FXR1-WT and KO macrophages. As shown in **Table 2B**, FXR1-KO macrophages produced higher cytokine/chemokine levels (IL-6, CCL2, and CCL5) than FXR1-WT cells following LPS stimulation, as expected. 4HPR treatment significantly inhibited LPS-induced IL-6 secretion by both FXR1-WT and KO macrophages in comparison to cells stimulated with LPS alone (*p*<0.001 for both cell lines; **Table 2B**). The 4HPR drug treatment reduced CCL2 levels in LPS-stimulated FXR1-WT cells (*p*<0.001). Interestingly, basal secretion of CCL2 was detectable and the 4HPR treatment was able to decrease basal secretion of CCL2 in WT macrophages (*p*<0.001; Table 2A). No significant effects of 4HPR were observed on basal secretion of CCL2 in FXR1-KO macrophages. Conversely, 4HPR treatment significantly decreased LPS-induced CCL5 production by both FXR1-WT (*p* = 0.001) and FXR1-KO (*p* = 0.002) macrophages.

**Table 2:** Effect of 4HPR or ERK inhibitor (UO126) treatment on cytokine secretion in FXR1-WT & KO macrophage cell lines.

A		Medium	4HPR	*p* value^a^	UO126^b^	*p* value^a^
		*n = 8*	*n = 8*	(4HPR vs Medium)	*n = 4*	(UO126 vs Medium)
**IL-6** (pg/ml)	**FXR1-WT**	0.0±0.0	0.0±0.0	= 0.721	0.0±0.0	= 0.808
	**FXR1-KO**	0.0±0.0	0.0±0.0	= 0.721	0.0±0.0	= 0.808
**CCL2** (pg/ml)	**FXR1-WT**	64.9±5.2	32.6±4.5	**<0.001**	24.5±8.4	** = 0.002**
	**FXR1-KO**	214.3±24.5	170.6±19.8	= 0.187	194.5±29.3	= 0.637
**CCL5** (pg/ml)	**FXR1-WT**	1.0±0.7	4.8±1.0	= 0.136	2.5±1.4	= 0.808
	**FXR1-KO**	6.5±1.9	8.0±1.4	= 0.521	2.5±1.4	= 0.203

B		LPS	LPS & 4HPR	*p* value^a^	LPS & UO126^b^	*p* value^a^
		*n = 12*	*n = 12*	(LPS & 4HPR vs LPS)	*n = 4*	(LPS & UO126 vs LPS)
**IL-6** (pg/ml)	**FXR1-WT**	225.5±29.0	36.5±5.6	**<0.001**	85.0±10.6	** = 0.034**
	**FXR1-KO**	1877.8±177.8	931.4±96.2	**<0.001**	758.0±52.2	** = 0.006**
**CCL2** (pg/ml)	**FXR1-WT**	482.3±52.6	106.4±9.8	**<0.001**	193.5±6.5	** = 0.004**
	**FXR1-KO**	2409.6±180.6	2011.0±228.6	= 0.185	2394.8±176.5	= 0.965
**CCL5** (pg/ml)	**FXR1-WT**	221.7±18.9	136.1±13.4	** = 0.001**	128.8±13.5	** = 0.011**
	**FXR1-KO**	732.8±55.8	402.9±45.1	** = 0.002**	500.8±29.4	** = 0.009**

a The *p* values were calculated using unpaired *t*-test.

b ERK inhibitor UO126 used at 5 µM.

The article "Fenretinide Corrects the Imbalance between Omega-6 to Omega-3 Polyunsaturated Fatty Acids and Inhibits Macrophage Inflammatory Mediators via the ERK Pathway" was published in 2013. Journal: PLoS One.

Next, we wanted to test the biological importance of ERK1/2 phosphorylation in these two cell lines. We have chosen to test CCL2 because basal levels of this chemokine are detectable, thus activation of ERK1/2 by external stimuli, such as LPS, would not be a factor in assessing its biological relevance. Furthermore, as shown in **Table 2A**, FXR1-KO cells, which have more phosphorylation of ERK1/2, express approximately 3 times higher levels of CCL2 (*p*<0.01) without stimulation by LPS when compared with WT macrophages. Therefore, we assessed whether inhibiting the phosphorylation of ERK1/2 could reduce CCL2 expression and whether the difference in its expression between KO and WT macrophages would be affected.

As we had observed with fenretinide, the UO126 ERK1/2 inhibitor was able to diminish the expression of CCL2 in WT cells (*p* = 0.002; **Table 2A**) but not in KO cells thus the difference between KO and WT macrophages in CCL2 secretion remained. FXR1-dependent modulation of CCL2 by both fenretinide and ERK1/2 inhibitors suggest that FXR1 protein might be particularly important in the posttranscriptional regulation of this particular chemokine.

We also tested the effects of UO126 ERK1/2 inhibitor on LPS-induced IL-6, CCL2, and CCL5 gene expression. The treatment of both LPS-stimulated FXR1-WT and KO macrophages with the ERK1/2 inhibitor resulted in a reduction of IL-6 protein (*p* = 0.034 and *p* = 0.006 respectively; **Table 2B**), and CCL5 protein (*p* = 0.011 and *p* = 0.009 respectively; **Table 2B**). CCL2 protein levels were reduced in FXR1-WT macrophages treated with the ERK1/2 inhibitor UO126 (*p* = 0.004) but not in KO macrophages (*p* = 0.965, **Table 2B**). The difference in IL-6, CCL2, and CCL5 protein expression was still present between LPS-stimulated FXR1-WT and KO macrophages treated with UO126 (*p*<0.001 for all three proteins). The inflammatory cytokine expression patterns in macrophages treated with the ERK1/2 inhibitor were very similar to the patterns observed between WT and KO macrophages treated with 4HPR. Therefore, it seems that fenretinide and ERK1/2 inhibitor share similar effects on the phosphorylation of ERK1/2 and on their ability to inhibit the expression of inflammatory proteins.

The article "Fenretinide Corrects the Imbalance between Omega-6 to Omega-3 Polyunsaturated Fatty Acids and Inhibits Macrophage Inflammatory Mediators via the ERK Pathway" was published in 2013. Journal: PLoS One.

### Fatty Acid Profiles in FXR1-KO and WT Macrophages

In the next series of experiments, we investigated the role of the two specific polyunsaturated omega-3 and omega-6 fatty acids in the excessive phosphorylation of ERK1/2 protein observed in FXR1-KO macrophages. Specifically, we measured the levels of two important phospholipid-esterified fatty acids, the pro-inflammatory arachidonic acid (AA) and the anti-inflammatory docosahexaenoic acid (DHA) in lysates prepared from unstimulated and LPS-stimulated FXR1-WT and FXR1-KO macrophages. The AA/DHA ratios derived from absolute AA and DHA levels were also calculated. The levels of nitrotyrosine and malonyldealdehyde, two oxidative stress indicators, were quantified as well.

We found significantly higher AA levels in LPS-stimulated FXR1-WT (*p*<0.001; **Fig. 3A**) and FXR1-KO macrophages (*p*<0.001; **Fig. 3B**) compared with unstimulated cells (medium). Also after LPS stimulation, DHA levels were significantly lower in FXR1-KO macrophages (*p* = 0.044; **Fig. 3D**) but not in FXR1-WT macrophages (*p* = 0.163; **Fig. 3C** **)** versus unstimulated cells. Increased AA/DHA ratios associated with LPS stimulation was observed in both FXR1-WT (*p* = 0.038; **Fig. 3E**) and FXR1-KO macrophages (*p*<0.001; **Fig. 3F**). A tendency was observed in LPS-stimulated FXR1-KO macrophages to have higher levels of AA than WT macrophages but a statistically significant difference was not reached. However, a significant reduction of DHA was observed in lipopolysaccharide-stimulated FXR1-KO macrophages when compared with WT cells (*p* = 0.041). Consequently, the AA/DHA ratio was significantly higher in FXR1-KO cells compared with FXR1-WT cells stimulated with LPS (*p*<0.001).

**Figure 3:** 4HPR treatment of LPS-stimulated FXR1-KO macrophage restores phospholipid-esterified fatty acids level to basal level. FXR1-WT (▪) and FXR1-KO (□) macrophages (50×10^6^ cells) were untreated or pre-treated with 4HPR (0.625 µM) for 21 h and then unstimulated or stimulated for 3 h with LPS (50 ng/ml). Cells were harvested and resuspended in BHA solution. (A) and (B) AA levels in FXR1-WT and KO macrophages respectively; (C) and (D) DHA levels; (E) and (F) AA:DHA ratios. Results are presented as mean ± SEM of four independent experiments. Differences were analyzed by one way ANOVA followed by a Student-Newman-Keuls secondary analysis, and were considered to be significant at *p*≤0.05. * indicates *p*<0.05.

### Fenretinide Treatment Restores AA/DHA Balance in LPS-Stimulated FXR1-KO and WT Macrophages

Previous studies in our laboratory demonstrated that cystic fibrosis mice with a chronic inflammatory lung disorder have higher levels of AA and lower levels of DHA. Moreover, we recently reported that treatment with 4HPR *in vivo* was able to correct this systemic defect in the CF mice [19], [20]. Therefore, we decided to investigate if treatment with 4HPR *in vitro* can also correct the low levels of DHA and high levels of AA observed in LPS-stimulated macrophages to the levels seen in unstimulated cells. 4HPR treatment completely reverted the LPS-induced increases in AA levels in both FXR1-WT (*p*<0.003) and FXR1-KO (*p*<0.001) macrophages (**Fig. 3A–B**). 4HPR treatment did not significantly modulate DHA levels in LPS-stimulated macrophages (**Fig. 3C–D**). However, 4HPR treatment significantly decreased AA/DHA ratios in LPS-stimulated FXR1-WT (*p* = 0.019) and FXR1-KO (*p* = 0.001) macrophages compared with LPS-stimulated cells (**Fig. 3E–F**). We also analyzed the effect of 4HPR treatment prior to stimulation with LPS on phospholipid-bound fatty acid levels. As shown in **Fig. 3C–D**, 4HPR treatment increased DHA levels in both FXR1-WT and KO macrophages compared with untreated macrophages (Medium), but no significant effects on AA levels were observed. These results demonstrate that the balance between phospholipid-bound AA and DHA might play an important role in the regulation of inflammatory AU-rich genes modulated by FXR1 RNA-binding protein.

The article "Fenretinide Corrects the Imbalance between Omega-6 to Omega-3 Polyunsaturated Fatty Acids and Inhibits Macrophage Inflammatory Mediators via the ERK Pathway" was published in 2013. Journal: PLoS One.

It is well documented that activating macrophages with LPS induces several oxidative processes [35]. Therefore, it was important to test if there were any differences in the lipid oxidation state that might account for the divergent AA/DHA ratios between FXR1-KO and WT macrophages. Our results suggest that the defects observed in phospholipid-bound fatty acid levels in FXR1-KO macrophages as compared to WT macrophages cannot be explained by aberrant oxidation in FXR1-KO cells. We did not find significant differences in the levels of nitrotyrosine and malonyldealdehyde between these two macrophage cell lines under unstimulated or LPS-stimulated conditions (**Fig. 4A–B**). As expected, activation of macrophages with LPS induced levels of both markers of oxidation in both FXR1-WT and KO macrophages. Interestingly, 4HPR treatment was able to reduce the effect of LPS on the levels of these two markers, leveraging them to pre-activated state levels (**Fig. 4A–B**). This test was done to exclude the possibility that differences in the lipid oxidation state might account for the divergent AA/DHA ratios between FXR1-KO and WT macrophages. No such differences were found. These results therefore exclude the oxidation of lipids as a possible mechanism responsible for the aberrant AA/DHA ratio in FXR1-KO compared to FXR1-WT macrophages. However, an effect of nitrotyrosine on activation of ERK1/2 cannot be excluded but since no differences between FXR1-KO and WT were found, differences on AA/DHA ratios are unlikely caused by lipid oxidation.

The article "Fenretinide Corrects the Imbalance between Omega-6 to Omega-3 Polyunsaturated Fatty Acids and Inhibits Macrophage Inflammatory Mediators via the ERK Pathway" was published in 2013. Journal: PLoS One.

**Figure 4:** Oxidative stress analysis of FXR1-WT and KO macrophage cell lines stimulated with the TLR4-ligand LPS. FXR1-WT (▪) and FXR1-KO (□) macrophages (50×10^6^ cells) were untreated or pre-treated with 4HPR (0.625 µM) for 21 h and then unstimulated or stimulated for 3 h with LPS (50 ng/ml). Cells were harvested and resuspended in BHA solution. (A) Nitrotyrosine levels and (B) Malonyldealdehyde levels in FXR1-WT and KO macrophages; Results are presented as mean ± SEM of four independent experiments. Differences were analyzed by one way ANOVA followed by a Student-Newman-Keuls secondary analysis, and were considered to be significant at *p*≤0.05. * indicates *p*<0.05.

Next, we tested the addition of exogenous AA or DHA on macrophages in order to verify their impact on endogenous AA and DHA phospholipid-bound levels. As shown in **Fig. 5A**, treatment of macrophages with AA increased endogenous AA and reduced DHA levels in macrophages. Inversely, the treatment of macrophages with DHA reduced AA and increased DHA, resulting in an important decrease of the AA/DHA ratio when compared to untreated macrophages (*p*<0.001; **Fig. 5C**). These data demonstrate the importance of the relative levels of AA versus DHA on the overall metabolism of these two phospholipid-esterified fatty acids and on their ratio in macrophages.

**Figure 5:** Interactions between AA and DHA in macrophage cell lines stimulated with exogenous AA or DHA. FXR1-WT (▪) macrophages (50×10^6^ cells) were treated with either arachidonic acid (100 nM) or docosahexaenoic acid (100 nM) for 21 h. Cell were harvested and resuspended in BHA solution. (A) AA levels in FXR1-WT macrophages; (B) DHA levels; (C) AA:DHA ratios. Results are presented as mean ± SEM of four independent experiments. Differences were analyzed by one way ANOVA followed by a Student-Newman-Keuls secondary analysis, and were considered to be significant at *p*≤0.05. * indicates *p*<0.05.

### AA and DHA Modulate Phosphorylation of ERK1/2 in Both FXR1-WT and KO Macrophages

Since FXR1-KO macrophages had higher AA/DHA ratios compared to FXR1-WT macrophages and also displayed higher phosphorylation of ERK1/2 than FXR1-WT macrophages, we then tested if the addition of exogenous AA and DHA might directly affect the phosphorylation of ERK1/2.

The article "Fenretinide Corrects the Imbalance between Omega-6 to Omega-3 Polyunsaturated Fatty Acids and Inhibits Macrophage Inflammatory Mediators via the ERK Pathway" was published in 2013. Journal: PLoS One.

As shown in **Fig. 6**, AA-treated FXR1-WT (**Fig. 6A**) and FXR1-KO macrophages (**Fig. 6B**) had statistically significant higher levels of ERK1/2 phosphorylation when compared to corresponding untreated cells. The addition of either U0126 ERK1/2 inhibitor or PD98059 ERK1/2 inhibitor to FXR1-WT or FXR1-KO macrophages treated with AA resulted in a dramatic reduction of ERK1/2 phosphorylation.

**Figure 6:** AA and DHA modulate phosphorylation of ERK1/2 in both FXR1-WT and KO macrophages. FXR1-WT (A and C) and FXR1-KO (B and D) macrophage cell lines (1×10^6^ cells) were untreated (Medium) or treated with AA (100 nM) or DHA (100 nM) for 21 h. ERK1/2 inhibitors (UO126 or PD98059) (5 µM) were added 60 min prior to harvesting where indicated and LPS (50 ng/mL) was added for 30 min where indicated. Cells were harvested and levels of phospho-ERK1/2 and total ERK1/2 MAPK in FXR1-WT and KO cells were analyzed by Western Blot. Total corresponding protein levels (ERK1/2) were used to normalize differences in loading. (A) and (B) AA increased ERK 1/2 phosphorylation in both FXR1-WT (A) and FXR1-KO (B) macrophages. (C) and (D) DHA decreased ERK 1/2 phosphorylation in both FXR1-WT (C) and FXR1-KO (D) macrophages. DHA also decreased phosphorylation after LPS stimulation in both cell types. As expected, ERK1/2 inhibitors resulted in the inhibition of ERK1/2 phosphorylation in both FXR1-WT and FXR1-KO macrophages. Results are presented as mean ± SEM of four independent experiments. Differences were analyzed by one way ANOVA followed by a Student-Newman-Keuls secondary analysis, and were considered to be significant at *p*≤0.05. * indicates *p*<0.05.

The effect of treatment using exogenous DHA on the phosphorylation of ERK1/2 in both FXR1-KO and FXR1-WT macrophages was also analyzed. As shown in **Fig. 6**, DHA treatment resulted in a reduction of ERK1/2 phosphorylation in both FXR1-WT (**Fig. 6C**) and FXR1-KO (**Fig. 6D**) macrophages compared to the ERK1/2 phosphorylation levels detected in untreated macrophages. Moreover, addition of either UO126 or PD98059 ERK1/2 inhibitors to DHA-treated macrophages resulted in even further reduction of ERK1/2 phosphorylation.

We have also tested if the DHA treatment was able to prevent the LPS induced ERK1/2 phosphorylation in both macrophage cell lines. Indeed, when either FXR1-WT or FXR1-KO macrophages were treated with LPS in the presence of DHA, no induction by LPS of ERK1/2 phosphorylation was observed (**Fig. 6C, 6D**). The DHA treatment was able to bring the levels of ERK1/2 phosphorylation to the levels observed in untreated macrophages. The treatment of macrophages with either UO126 ERK inhibitor or PD98059 ERK1/2 inhibitor led to further inhibition of ERK1/2 phosphorylation in LPS treated FXR-WT and FXR1-KO macrophages.

The article "Fenretinide Corrects the Imbalance between Omega-6 to Omega-3 Polyunsaturated Fatty Acids and Inhibits Macrophage Inflammatory Mediators via the ERK Pathway" was published in 2013. Journal: PLoS One.

Next, we verified if the modulation of ERK1/2 phosphorylation by AA or DHA had a biological relevance. The elevated phosphorylation of ERK1/2 is associated with augmented expression of inflammatory cytokine and chemokine genes [36]. The treatment of both FXR1-WT and KO macrophages with AA lead to a statistically significant increase of IL-6, CCL2, CCL5 (**Fig. 7**), and TNF (**Fig. 8**) secretion when compared to untreated macrophages. Inversely, the reduction of ERK1/2 phosphorylation by DHA resulted in the reduction of IL-6, CCL2, CCL5 (**Fig. 7**), and TNF (**Fig. 8**) secretion in LPS-stimulated macrophages. Furthermore, treatment of AA-stimulated macrophages with UO126 ERK1/2 inhibitor (5 µM) reduced TNF to almost basal levels in both FXR1-WT and KO macrophages, as shown in **Fig. 8**.

**Figure 7:** Biological effect of the modulation of ERK1/2 phosphorylation by AA or DHA on cytokines and chemokines gene expression. FXR1-WT (▪) and FXR1-KO (□) macrophage cell lines (2.5×10^5^ cells) were untreated (Medium) or treated with AA (100 nM) or DHA (100 nM) for 21 h. Cells were also stimulated with 50 ng/ml of LPS for 3 h. Cell supernatants were harvested and levels of IL-6 (A), CCL2 (B), and CCL5 (C) were analyzed by Luminex platform assay. Results are presented as mean ± SEM of three independent experiments. Differences were analyzed using an unpaired *t*-test and were considered to be significant at *p*≤0.05. * indicates *p*<0.05.

**Figure 8:** Biological effect of the modulation of ERK1/2 phosphorylation by AA or DHA on TNF gene expression. FXR1-WT (▪) and FXR1-KO (□) macrophage cell lines (2.5×10^5^ cells) were untreated (Medium) or treated with AA (100 nM) or DHA (100 nM) for 21 h. Cells were also treated with the ERK1/2 inhibitor UO126 (5 µM) concurrently with the AA treatment or stimulated with 50 ng/ml of LPS for 3 h where indicated. Cell supernatants were harvested and levels of TNF were analyzed by ELISA. Results are presented as mean ± SEM of three independent experiments. Differences were analyzed using an unpaired *t*-test and were considered to be significant at *p*≤0.05. * indicates *p*<0.05.

Overall, our results demonstrate the importance of the balance in fatty acids in the regulation of expression of inflammatory genes. They show the powerful normalizing effect of 4HPR on the deregulated inflammation observed in macrophages with ablated *Fxr1* gene encoding an important AU-rich binding protein which regulates translational repression of inflammatory genes.

## Discussion

Our previous studies demonstrated that FXR1 is able to negatively regulate TNF gene expression at the post-transcriptional level [8]. We also showed that FXR1 ablation triggers elevated expression of other inflammatory cytokines and chemokines in macrophage cell lines following stimulation with LPS [30]. RNA-binding proteins play a key role in the post-transcriptional regulation of inflammatory cytokines by regulating mRNA translation, mRNA stability, and mRNA nuclear export [14], [37]–[41]. In turn, the activity of many RNA binding proteins is regulated by several kinases, including MAP kinases.

The article "Fenretinide Corrects the Imbalance between Omega-6 to Omega-3 Polyunsaturated Fatty Acids and Inhibits Macrophage Inflammatory Mediators via the ERK Pathway" was published in 2013. Journal: PLoS One.

MAP kinases are expressed constitutively but must undergo activation before they can exert their functional activity. Upon ligation of TLRs by ligands such as LPS, MAP kinases become activated and subsequently transmit intracellular signals that result in macrophage activation and cytokine gene expression. Both ERK1/2 and p38 MAPK signaling pathways have been implicated in the regulation of cytokine gene expression by modulating both transcriptional and post-transcriptional processes [13], [40]. The post-transcriptional regulation of cytokines such as TNF may involve multiple RNA binding proteins, including TTP, HuR, TIA-1, TIAR, and FXR1 protein [6]–[8], [30]. p38 MAPK, acting through the downstream kinase MK2, can modulate the expression of TTP at the transcriptional and post-translational level. These events in turn will destabilize TNF mRNA in an ARE-dependent manner [14]. Our results presented here show that ERK1/2 MAP kinase but not p38 MAP kinase is over-activated in unstimulated and LPS-stimulated FXR1-KO macrophage cell lines compared with FXR1-WT macrophages. ERK1/2 is also able to phosphorylate TTP and is involved in TTP-mediated regulation of TNF mRNA stability [42].

Recent data show that TTP regulation requires the combined action of both ERK and p38 MAPK pathways [15], [43]. With ablation of FXR1, cells exhibit over-activation of ERK1/2 and much higher gene expression of TNF and other proinflammatory cytokines and chemokines. We previously showed that TNF mRNA stability and steady state levels are not affected by the absence of FXR1 [8], [30]. As TTP is known for its role in destabilizing TNF mRNA, the effect of over-activated ERK1/2 on increased TNF gene expression in LPS-stimulated FXR1-KO macrophages likely cannot be explained by the effect of FXR1 ablation on the regulatory activity of TTP. Therefore, it is more likely that many other downstream proteins phosphorylated by ERK1/2 are involved. One possible candidate is ribosomal protein S6 kinase, which can activate eukaryotic translation initiation factor 4B [44]. This would lead to enhanced translatability of TNF mRNA and consequently higher gene expression of this inflammatory cytokine. As a result, FXR1 might exert strong repressive activity via two possible mechanisms: one as a translational repressor of TNF mRNA [8] and the other by controlling the activity of ERK1/2.

The article "Fenretinide Corrects the Imbalance between Omega-6 to Omega-3 Polyunsaturated Fatty Acids and Inhibits Macrophage Inflammatory Mediators via the ERK Pathway" was published in 2013. Journal: PLoS One.

Lo and colleagues demonstrated that MAP kinases can be regulated by alterations in phospholipid-bound fatty acid metabolism [16]. In this study, we performed a detailed analysis of phospholipid-bound fatty acid levels in unstimulated and LPS-stimulated FXR1-WT and KO macrophage cell lines. Our results showed that the ablation of FXR1 resulted in augmented ratios of AA/DHA in LPS-stimulated macrophages. More specifically, after LPS stimulation, FXR1-KO macrophages had diminished DHA levels and higher AA/DHA ratios compared with FXR1-WT macrophages. These altered lipid profiles were associated with enhanced phosphorylation of ERK1/2. This association was confirmed by the increase of ERK1/2 phosphorylation in macrophages following their treatment with AA while the treatment with DHA resulted in a reduction in ERK1/2 phosphorylation. This is in accordance with recent reports which show that DHA is able to downmodulate ERK1/2 activation [45], [46].

Unstimulated FXR1-KO macrophages can secrete higher levels of the chemokine CCL2 at baseline than their WT counterparts. However, the overall concentration of this mediator is fairly low, most likely too low to impair phospholipid homeostasis in these cells. Indeed, the AA/DHA ratio is not significantly different between non-activated WT and KO macrophages. Once the macrophages are stimulated with LPS, the concentration of inflammatory cytokines and oxidative stress markers becomes dramatically higher in FXR1-KO than WT macrophages, resulting in the degradation of more sensitive species of phospholipids such as DHA in FXR1-KO cells. This decrease in DHA levels in FXR1-KO macrophages might have reduced their control of further inflammatory cascades in response to LPS since DHA has anti-inflammatory properties [47], [48]. Furthermore, we demonstrated that DHA and AA relative levels are closely related and a decrease in DHA leads to an increase of AA levels. Therefore, the outcome of this increased AA/DHA ratio results in a higher phosphorylation of ERK1/2, which has a direct effect on the increased expression of inflammatory mediators.

We previously reported lower levels of several cytokines in 4HPR-treated animals [20]. Similarly, Vilela and colleagues showed that mutant *Cftr* human tracheal epithelial cells produce much less IL-8 after stimulation with TNF when these cells are pre-treated with 4HPR [49]. The results of the present study demonstrate that the treatment of macrophages with 4HPR induces anti-inflammatory effects. 4HPR was able to lower the expression of TNF as well as other cytokines (IL-6) and chemokines (CCL2 and CCL5). It has been previously demonstrated that 4HPR-induced apoptosis of neuroblastoma [50] and head and neck squamous carcinoma cells involves activation of both p38 MAPK and ERK1/2 MAPK [51], [52]. Therefore, we also assessed the phosphorylation of these two important kinases. Our results showed that ERK1/2 MAPK was over-phosphorylated in FXR1-KO macrophages while p38 MAPK phosphorylation did not vary between FXR1-KO and WT macrophages. Moreover, treatment with 4HPR reduced the phosphorylation of ERK1/2 MAPK without modifying p38 MAPK phosphorylation status in both FXR1-KO and WT macrophages. However, the restoration of LPS-induced ERK1/2 MAPK phosphorylation to basal levels by 4HPR was associated with a downregulation (without complete elimination) of the expression of TNF protein and other inflammatory cytokines and chemokines.

The article "Fenretinide Corrects the Imbalance between Omega-6 to Omega-3 Polyunsaturated Fatty Acids and Inhibits Macrophage Inflammatory Mediators via the ERK Pathway" was published in 2013. Journal: PLoS One.

Based on our results, we do not see an effect of FXR deletions on the levels of PUFA at baseline. It is unlikely that there is a direct link between FXR and the regulation of PUFA. However, the ablation of FXR creates a greater inflammatory response to LPS stimulation which can be normalized with 4HPR, through increases in DHA. In fact, DHA was shown to act as an inhibitor of various TLRs and TLR mediated signaling pathways, including ERK1/2 [46]. Thus, 4HPR affecting DHA levels may explain why we observe the downregulation of ERK1/2 activation, ultimately resulting in the downregulation of TNF expression. These results indicate that other signaling pathways remained active in 4HPR-treated macrophages, suggesting that 4HPR selectively affects specific regulatory pathways without a generalized shutdown of signaling mechanisms in LPS-activated macrophages. This regulatory effect of 4HPR on macrophages secretion of inflammatory cytokines might be one reason why this agent has been used successfully as adjuvant therapy in cancer and recently also in inflammatory diseases.

Our proposed model of action of 4HPR in modulating the expression of inflammatory mediators that are deregulated in FXR1-ablated macrophages is shown in **Fig. 9A and 9B**. The initial augmentation of gene expression in LPS-activated FXR1-KO macrophages is much higher than observed in WT macrophages. 4HPR inhibition of inflammatory gene expression in FXR1-KO macrophages is less efficient than in FXR1-WT macrophages due to ablation of this important regulatory gene. FXR1 is an RNA-binding protein that negatively regulates inflammatory genes in a post-transcriptional manner [8], [30]. Non-activated macrophages that have the *Fxr1* gene ablated have an increase of ERK1/2 phosphorylation and an increase in the expression of some AU-rich genes such as CCL2. Treatment of these macrophages with 4HPR raises the level of DHA, which we showed to diminish the phosphorylation of ERK1/2. Therefore, a subsequent reduction of the expression of certain AU-rich genes such as CCL2 occurs, as observed. LPS stimulation activates these macrophages by triggering MAPK pathways, including ERK1/2 MAPK. The augmentation of ERK1/2 phosphorylation results in an increase of the expression of many inflammatory mediators such as TNF, IL-6, CCL2, and CCL5. The higher expression of these inflammatory mediators in FXR1-KO than WT macrophages is accompanied by a significant reduction in DHA and a slight increase in AA that leads to a higher AA/DHA ratio imbalance in FXR1-KO macrophages. We showed that an increase in the levels of AA is able to further increase the phosphorylation of ERK1/2, which results in a positive feedback loop for the production of more inflammatory mediators. Fenretinide is able to keep the generation of inflammatory mediators under control by modifying the lipid imbalance, directing it towards an anti-inflammatory state by diminishing the AA/DHA ratio. This results in a reduction in the phosphorylation of ERK1/2 leading to a diminution of inflammatory cytokine genes expression, which we observed in this study.

The article "Fenretinide Corrects the Imbalance between Omega-6 to Omega-3 Polyunsaturated Fatty Acids and Inhibits Macrophage Inflammatory Mediators via the ERK Pathway" was published in 2013. Journal: PLoS One.

**Figure 9:** Fenretinide – a key player in reducing the expression of inflammatory genes. (A) In non-activated macrophages treatment with fenretinide can reduce constitutive expression of AU-rich genes such as CCL2 by augmenting the DHA levels in non-activated macrophages. This results in a lowering of ERK1/2 phosphorylation leading to a diminution in the expression of certain constitutively inflammatory genes. (B) In LPS- activated macrophages, treatment with fenretinide exerts its anti-inflammatory role by reducing the AA/DHA ratio that is increased by activation of macrophages with various stimuli, including LPS, a TLR4 ligand. This lowers ERK1/2 phosphorylation, which results in a reduction of the expression of several inflammatory genes.

Overall, our results provide insight into the possible mechanisms underlying the model of action of 4HPR and demonstrate an important molecular link between the regulation of inflammatory cytokine/chemokine expression and fatty acid composition in macrophages following activation by endotoxins.
